# Metabolite Comparison between Spleen-Deficiency and Healthy Children

**DOI:** 10.1155/2023/5937308

**Published:** 2023-04-12

**Authors:** Zhiyi Liang, Qianzeng Fu, Haiman Li, Xuan Xu, Panting Ding, Wei Tang, Yong Ye, Xiangning Shao, Xiaowen Tan, Xiaojun Wang, Xun Luo, Jun Wang, Dejun Wang, Huan Zhong, Mi Liu

**Affiliations:** ^1^School of Acupuncture-Moxibustion, Tuina and Rehabilitation, Hunan University of Chinese Medicine, Changsha 410208, China; ^2^Hunan Acupuncture & Moxibustion, Clinical Medicine Research Center, The First Hospital of Hunan University of Chinese Medicine, Changsha 410007, China; ^3^Xiangxi Hospital of Chinese Medicine of Tujia and Miao Ethnic Group, Jishou 416000, China; ^4^Kerry Rehabilitation Medicine Research Institute, Shenzhen 518000, China; ^5^Department of Anatomy, School of Medicine, Shenzhen University, Shenzhen 518060, China

## Abstract

**Objective:**

From the perspective of metabolomics, this study compares the metabolomics characteristics of feces and urine between children with spleen-deficiency and healthy children to explain the scientific connotation of children with spleen-deficiency susceptibility to digestive system diseases from the metabolic level and provide a scientific basis for further research.

**Methods:**

This study included 20 children with spleen-deficiencies and 17 healthy children. Children's symptom scores, height, and weight were recorded in groups, and feces and urine samples were collected. The samples were detected using ultrahigh-performance liquid chromatography-mass spectrometry. The data were analyzed using multivariate statistical analysis such as principal component analysis (PCA) and partial least squares discriminant analysis (PLS-DA). Related differential metabolites were identified through database comparisons between two groups based on the MS and KEGG.

**Results:**

Compared to healthy children, the metabolites glucuronic acid, xanthine, and indole-3-acetaldehyde tend to be reduced in children with spleen-deficiency. Moreover, these children showed an increase in metabolites such as quinic acid, adenine, 4-methyl-5-thiazole-ethanol, 3-formyl indole, and 5-hydroxy indole-3-acetic acid. The condition affected many of the critical metabolic pathways, including the metabolism of tryptophan, cysteine, methionine, and pentose phosphate.

**Conclusion:**

The children with spleen-deficiency had disorders at the metabolic level, which might be due to factors such as diet, personal preferences, and genes, leading to various symptoms, making spleen-deficiency children more prone to suffer from digestive diseases than healthy children. The results set a basis for the research on children's TCM constitution, which can be a reference to further studies to deal with the spleen-deficiency.

## 1. Introduction

People have different characteristics of suffering from the same disease due to various classifications such as gender, race, and region [1–4]. For instance [3], researchers found that MS-specific mortality trends demonstrate distinctive disparities by race/ethnicity and age. In traditional Chinese medicine (TCM) [5], there is also a kind of classification approach called constitution classification, which has similar functions to those classifications mentioned above but only different names. Dong's team had attempted to help the theory of the TCM constitution move towards internationalization in the translation of the academic term, and names will not affect the connotation of the classification methods [6].

A TCM constitution refers to the comprehensive and relatively stable inherent characteristics of the human body in terms of morphological structure, physiological function, and psychological state that are formed based on the innate and acquired endowment [7]. The TCM constitution is the internal basis of disease occurrence, development, transformation, and prognosis. TCM doctors can diagnose a person's constitution by identifying patterns and then infer their potential disease spectrum by analyzing the constitution, even if the patient is not “sick” as per modern diagnostic techniques [8].

People with the exact constitution have similar susceptibilities to certain diseases. Liang's team [4] preliminarily revealed the correlation between constitution and diseases in 1639 studies in 2020. A report showed the relationship between allergic rhinitis and constitution in 2022 [9]. And in 2021, a cross-sectional study demonstrated the association of constitution and female patients with systemic lupus erythematosus [10]. More and more research on the TCM constitution show that targeted treatments for people with different constitution types will help reduce the risk of suffering from certain diseases.

The constitution analyses also apply to children even if there is no targeted standard of the TCM constitution for them [11, 12]. However, there is not much international research about children on the TCM constitution. Since children with spleen-deficiency account for much of children's constitution classification, we chose this constitution as our objective [13]. These children normally have symptoms like emaciation, listlessness, fatigue, sweating, poor appetite, indigestion, muscle weakness, irregular stool, or even persistent diarrhea. Their growth and development are slower than those of healthy children (called balanced constitution in TCM), which easily affects the function of the digestive and other systems, making spleen-deficiency children more susceptible to digestive diseases [14–17]. For instance, spleen-deficiency may result in phlegm dampness, which can easily cause lung diseases such as cough and asthma [18]. Childhood body physique is the foundation of lifelong health, and the subhealth status of children with spleen-deficiency is associated with numerous families. Children's health is closely related to the socioeconomic status of the country and the nation; it is an urgent concern of parents and clinicians to ensure children's healthy growth and find a way to improve their spleen-deficiency constitution. Therefore, our research aimed to investigate the distinct indicators between spleendeficiency and healthy children.

Metabolomics can effectively reveal the essence of an organism's metabolism and accurately reflect the biological system's state by exploring micromolecular metabolites and metabolic pathway products, which have been used in TCM constitution research [19–21]. In 2018, Chen's team [22] found that differentially expressed miRNAs may partly explain the TCM constitution's distinct characteristics, showing an excellent research example. And there is no report on the microscopic characterization of spleen-deficiency in children, either domestically or internationally.

Thus, this study aims to reveal the characteristics of small molecular metabolites and metabolic pathway products in children with spleen-deficiency and provide new ideas for improving the physique of such children and preventing related diseases.

## 2. Materials and Methods

### 2.1. Sources and Grouping of Cases

Children in the spleen-deficiency group were enrolled from October 2019 to December 2020 in the Pediatric Tuina Department, the Pediatric Outpatient Department of the First Affiliated Hospital of Hunan University of Traditional Chinese Medicine, and the Pingdi Kindergarten of Yueyang City, aged between one and six years. The healthy group was the openly recruited children from Pingdi Kindergarten in Yueyang City who were in good condition per the physical examination. According to the TCM identification standard, 20 children with spleen-deficiencies and 17 healthy children were included. The process of the experiment and the symptom list of 20 spleen-deficiency children are as follows (see Figure 1 and Table 1). (The entire name is hidden in Table 1 for privacy concerns).

### 2.2. Ethics Committee Approval

The Medical Research Ethics Committee of the Xiangxi Hospital of Chinese Medicine of the Tujia and Miao Ethnic Group provided the approval. All the participants' parents signed an informed consent form, and all work was conducted by the Declaration of Helsinki (1964) during the process (Protocol Registry Number: 2019-No. 08)

### 2.3. Principal Reagents and Instruments

Methanol was purchased from Sigma–Aldrich (Shanghai) Trading Co., Ltd.; acetonitrile, formic acid, and ammonium formate were obtained from Merck, USA; L-glutamic Acid-^13^C^5^, ^15^N was acquired from CATO, USA; L-Phenylalanine-^13^C^6^, L-Methionine-^13^C^5^ were obtained from CDN, Inc., CAN.

Ultrahigh-performance liquid chromatography-mass spectrometer (Ultimate 3000), high-resolution mass spectrometer (Q-Exactive), chromatographic column (HSS T3 100 *∗* 2.1 mm 1.8 *μ*m, Waters), vortex mixer (xw-80A), water purifier (Milli-Q Gradient A10), high-speed refrigerated Centrifuge (EPPENDORF-5415R), and termovap sample concentrator (NDK200-2N) were used.

### 2.4. Sample Collection and Storage

#### 2.4.1. Feces

About 30 mg of fresh feces from the participants was collected in the morning, and the feces were placed in a cryopreservation tube. The sample was then brought to the laboratory at an ordinary temperature within 1 hour and stored in a refrigerator at −80°C.

#### 2.4.2. Urine

The midstream urine of the participants was collected in the morning using a disposable urine collection cup, and about 10 mL of urine was poured into a cryopreservation tube. The sample was then brought to the laboratory at an ordinary temperature within 1 hour and stored in a refrigerator at −80°C.

### 2.5. Sample Preparation

#### 2.5.1. Feces

First, the samples were thawed at 4°C and swirled for 30 min. Then, 10 mg of the samples were weighed, 1000 *μ*L of 1% formic acid/acetonitrile mixture was added after an ice bath, and 20 *μ*L of 1000 *μ*g/mL internal standard was added, swirled for 1 min, and allowed to stand for 10 min.

The sample was centrifuged at 4°C, 13000 rpm for 5 min, and 800 *μ*L of the supernatant was collected in a centrifuge tube and flushed with nitrogen. Then, 100 *μ*L of acetonitrile/water/formic acid (80 : 19 : 1, v/v/v) was added to re-dissolve the sample. The sample was centrifuged again under the same conditions as described above. Finally, 70 *μ*L of the supernatant was collected and tested.

#### 2.5.2. Urine

First, the samples were thawed at a temperature of 4°C. The samples were centrifuged at 4°C, 13000 rpm for 5 min. All supernatants were filtered with a 0.22 *μ*m aqueous phase filtration membrane. After that, 80 *μ*L was taken, and 20 *μ*L of 1000 *μ*L g/mL internal standard was added, swirled for 30 s and tested.

### 2.6. Liquid Chromatography-Mass Spectrometry (LC-MS/MS) Metabolomics Test

The positive ion mode mobile phase was an aqueous solution containing 0.1% formic acid (liquid A) and 100% methanol containing 0.1% formic acid (liquid B). In contrast, the negative ion mode mobile phase was an aqueous solution containing 10 mM ammonia formate (liquid A) and 95% methanol containing 10 mM ammonia formate (liquid B). The details are presented in Tables 2 and 3.

### 2.7. Case Selecting Criteria

#### 2.7.1. TCM Identification Standard

The Diagnostic Criteria of Spleen Deficiency Syndrome in Children published by the Pediatric Committee of the Chinese Society of Integrated Traditional and Western Medicine in 2007 [23] and the related description of children's biased constitution in Pediatric Massage [24] (the textbook of the 13^th^ Five-Year Plan of National Higher Education edited by Professor Liao Pindong in 2016) were used as TCM spleen-deficiency identification standard. The main indexes included were (1) diarrhea or incomplete defecation, (2) sallow yellow or wan complexion, (3) poor appetite, (4) emaciation or puffiness, (5) light or fat tongue with teeth marks and greasy coating. Secondary indexes were (1) dark around the eyes, (2) spontaneous sweating or hyperhidrosis, (3) finger-licking and salivation, (4) mild anemia, (5) mild edema, (6) opening eyes while sleeping, (7) abdominal discomfort, (8) limb weakness and fatigue, and (9) faint finger venules and a weak pulse.

If three main or two main indexes combined with two secondary indexes were met (at least) and the symptoms persisted for over three months, the condition was classified as spleen-deficiency.

Balanced constitution [25]: A balanced constitution was defined as follows: normally developing, well-proportioned, muscular, energetic, lively, flexible, quick-reacting children with peaceful sleep, warm limbs, a moist skin, dark hair, moist complexion, vivid eyes, even breathing, loud crying, a strong voice, moderate diet, normal defecation, a pale red throat, a pale red tongue, and a thin and white tongue coating. Children with a balanced constitution can tolerate frequent climate change more efficiently and have fewer illnesses and allergies than other children. In this essay, we use “healthy children” as pronouns.

#### 2.7.2. Inclusion Criteria

Children meeting the following criteria are as follows: (1) meeting the identification standard mentioned above for children's spleen-deficiency constitution and healthy children; (2) age range: 1––6 years, regardless of gender; and (3) parents of children ready to participate and sign the informed consent form voluntarily.

#### 2.7.3. Exclusion Criteria

The exclusion criteria are as follows: (1) skin with burns, scratches, scabies, trauma, fractures, and bone dislocation; (2) acute infectious diseases such as osteomyelitis, cellulitis, erysipelas, and bone tuberculosis; (3) bacillary dysentery, amoebic dysentery, and cholera; (4) severe systemic diseases such as a serious malignant tumor, heart disease, psychosis, and liver and kidney diseases; and (5) use of hormone drugs or other traditional Chinese and western medicines or immunomodulators in the last three months.

#### 2.7.4. Rejection Criteria

The participants who met the following criteria are as follows: (1) patients who were unable to adhere to the treatment during the disease because of accepting other treatment plans halfway, having an accident halfway, or quitting the treatment on their own; (2) those within incomplete observations data, poor compliance (parents or children), and those asking for withdrawal during the trial; and (3) spleen-deficiency participants who passed the screening and developed the condition but did not complete the observation period for four weeks for some reason (regarded as shedding cases).

### 2.8. Observation Indicators

#### 2.8.1. General Information

Changes in stool, complexion, sleep, diet, weight, height, and other clinical manifestations were documented in healthy children and children with spleen-deficiency. The height and weight were recorded according to the Reference Standard for Growth and Development of Children under 7 in China in 2009 [26] by the Department of Maternal and Child Health and Community Health, Ministry of Health. The CRF table was made according to the Diagnostics of Traditional Chinese Medicine, the 11^th^ Five-Year Plan of higher education textbook edited by Zhu [27], and the grading of spleen-deficiency symptoms was done following the Guiding Principles of Clinical Research of New Chinese Medicine promulgated in 2002 [28].

#### 2.8.2. Metabonomic Characteristics

Analysis of different metabolites and metabolic pathways were done.

### 2.9. Data Processing

#### 2.9.1. Major Procedure

Analysis Base File Converter was used to convert the original data into the general format (abf). The data were preprocessed for peak identification, automatic integration, and retention time correction using the MS-DIAL software platform. A visual matrix containing metabolite number, retention time, mass-to-charge ratio, metabolite name, ion mode, and peak area were obtained. Subsequently, the feature number of samples was screened to obtain a result containing peak quantitative results (within sample names, ms1 and ms2) and the visual matrix (including the relative quantification of peak areas).

The substances were characterized according to the data of ms2, and a variety of metabolites were identified by comparing them with the MS Bank database. The comparison of the database is qualitative and then relatively quantitative by peak area, and the comparison between samples is presented by data analysis. The qualitative indicator is that substances with a score above 0.7 will be displayed in the qualitative table.

Then the relationship between multiple and individual metabolic pathways was analyzed using graphical functions. Principal component analysis (PCA) and partial least squares analysis (PLS-DA) were used to acquire the corresponding scores and loading plots, and the results were analyzed and compared. VIP values were extracted from the partial least-square discriminant analysis score chart. Generally, variables with a VIP > 1 have significant differences. Using the significant differences to obtain the following results, such as heatmap analysis and metabolic enrichment analyses.

#### 2.9.2. Database Application

The MS Bank and the Kyoto Encyclopedia of Genes and Genomes Database (KEGG) were used to analyze the spectrum of positive and negative ion metabolites and the metabolic pathways involved. The names and functions of the metabolites were identified by consulting the China National Knowledge Infrastructure (CNKI) literature, the human metabolite database (https://www.hmdb.ca), and the Kyoto Encyclopedia of Genes and Genomes database (https://www.kegg.jp/).

#### 2.9.3. Data Normalization

During the research, we normalized the data to eliminate the analysis error caused by different sample concentrations. Firstly, add the internal standard in each sample when preparing (mentioned in 2.5. Sample preparation). Secondly, use lowess to process the fluctuating data to achieve data fitting and normalization. The data obtained were saved in an Excel file for analysis and processing.

#### 2.9.4. Other Data Analysis

Other data were collected and sorted in Excel, compared, and analyzed using SPSS 21.0. Statistical significance was set at *P* < 0.05. The measurement data were expressed by “mean standard deviation” ($\bar{x}\pm S$). When a normal distribution was met, the paired *t*-test was used. The rank-sum test was used when the normal distribution was not satisfied, and the chi-square test was employed to analyze the counting data.

## 3. Data and Results

### 3.1. Basic Information Comparison

The basic information comparison between the healthy and spleen-deficiency group can be seen in Table 4.

### 3.2. Specimen Test Results of Feces and Urine

There are some legends in the upper-right corner of Figures 2–6, “A” or “a” represents the feces or urine results of the spleen-deficiency group, and “C” or “c” represents the feces or urine results of the healthy group.

#### 3.2.1. Ion Map

The total ion flow graphs of all QC samples were superimposed. The spectrogram overlapped well, and the retention time and peak signal intensity fluctuated little, indicating that the instrument was in good condition during the whole sample analysis process, which was suitable for the detection and analysis of the project.

According to the LC-MS/MS condition in the research methods, sample data were collected, and the total ion current was determined, as displayed in Figure 2. The chromatogram indicated differences in the number and height of chromatographic peaks in the feces of each group in positive and negative ion modes. These indicated substantial metabolites differences in feces and urine between the spleen-deficiency and healthy groups, which can be further analyzed and compared.

#### 3.2.2. PCA Score Chart

PCA is an unsupervised learning model which plays an important role in data dimensionality reduction. There were 643 metabolites with significance, 286 for feces and 357 for urine; they were used to generate the PCA and PLS-DA models. It is a k-dimensional feature reconstructed based on the original n-dimensional part. Based on the ion maps, the PCA score chart could be drawn.

First, the data was normalized and transformed by the Pareto scaling method. Then a set of mutually orthogonal coordinate axes in sequence from the original data square was found, and the choice of new coordinate axes was closely related to the data itself. Among them, the first new coordinate axis was the direction with the most significant variance in the original data, the second new coordinate axis was the plane orthogonal to the first coordinate axis, and the third axis was the plane orthogonal to the first and second axes. And so on, we got *n* coordinate axes. We found that in the new coordinate axes obtained in this way, most of the variance was contained in the first *k* coordinate axes, and the variance in the last coordinate axes was almost zero. So, we ignored the rest of the coordinate axes and only kept the first *k* coordinate axes with the most significant variance. This procedure was equivalent to retaining only the dimension features that contain most variance, and ignoring the feature dimensions that contain almost zero variance to reduce the dimension of data features.

As depicted in Figure 3, each group of samples' metabolic profile was clear. The pink parts stand for the spleen-deficiency group and the green ones for the healthy group. The ellipse represents the 95% confidence interval of a group of samples. The figure showed partial conglomerations of the two groups of models in the positive and negative ion modes with a pretty reappearance. A specific separation between the two sample groups indicates a difference in sample metabolism. The result lays a foundation for understanding the differential metabolic characteristics of the two groups and then comparing and analyzing PLS-DA results between them.

#### 3.2.3. PLS-DA Score Chart

The PLS-DA is a statistical method related to the PCA. After the reducing of the dimension of data features, the PLS-DA model was established. It projected the predicted and observed variables into a new space by way of projection to establish regression analysis between group (Y) and metabolite (X). A linear regression model was found during the process, which was used to find the difference between groups and get differential metabolites. Then several kinds of figures were obtained.

In the PLS-DA score chart (see Figure 4), the pink parts stand for the spleen-deficiency group and the green ones for the healthy group. The discrete and clustered figures showed the reproducibility of the samples and the metabolic profile between the sample groups. That means models in the same group were similar, while the two groups showed different metabolism features. A clear separation of the two groups of samples can be seen in the score chart. The metabolic profiles of feces and urine of children with spleen-deficiency and healthy children demonstrated significantly separated features.

#### 3.2.4. Cross-Validation of PLS-DA

Cross-validation (CV) was used to evaluate the quality of the model. CV divided the sample data into two parts: the training set and the verification set. The training set was used to build the model, and the verification set was used to test the model. *R*^2^ is the accuracy of the model establishment. *Q*^2^ is the prediction accuracy of the model. The higher the *Q*^2^ and *R*^2^ are, the higher the model's quality and prediction ability are.

Figure 4 is the resulting diagram of the cross-validation of the PLS-DA model. The abscissa shows the number of components the model selects, and the ordinate shows the values of *R*^2^, *Q*^2^, and accuracy. Generally, the group with the highest *R*^2^ and *Q*^2^ values was assigned. As depicted in Figure 5, the model had qualified prediction ability and accuracy.

#### 3.2.5. VIP Diagram of PLS-DA

The VIP diagram of PLS-DA can help people understand the contribution of different groups to sample differentiation and the significance of variables. After the model establishing, the contribution of each variable could be observed. VIP values were extracted from the PLS-DA score chart. Generally, variables with a VIP > 1 have significant differences. The differential metabolites with most significance were selected to form the figures. As depicted in Figure 6, “A” or “a” represents the feces or urine results of the spleen-deficiency group, and “C” or “c” represents the feces or urine results of the healthy group. The horizontal coordinates in the coordinate system on the left side of the figure are the VIP values, the vertical coordinates are the differential metabolites, and the color coding on the right side reflects the high and low concentrations of this metabolite in the different groups. The higher the VIP value is, the more significant the contribution to sample differentiation. The VIP score of metabolites in Figure 6 was more than 1, contributing significantly to the differences in the samples. The VIP colors and figures of the groups were different, indicating significant differences in the metabolites in feces and urine samples between the two groups.

#### 3.2.6. Heatmap Analysis

The VIP diagram-obtained differential metabolites were further visualized using heatmap analysis to provide a more intuitive understanding of the differences and distribution of data. As shown in Figure 7, “A” or “a” represents the feces or urine results of the spleen-deficiency group, and “C” or “c” represents the feces or urine results of the healthy group. The color in each gird stood for various data. The distribution of metabolites in feces and urine samples varies significantly between spleen-deficiency and healthy children.

#### 3.2.7. Differences in Metabolites of Feces and Urine

According to the metabolites (including positive and negative ions) with VIP > 1 in PLS-DA data results, many metabolites required further screening. Through *P* < 0.05 and FD > 1.5 or <0.75, it was found that there were three metabolites in the positive ion mode and five metabolites in the negative ion mode. Among them, glucuronic acid, xanthine, and indole-3-acetaldehyde indicated a downward trend, whereas quinic acid, adenine, 4-methyl-5-thiazole-ethanol, 3-formyl indole, and 5-hydroxy indole-3-acetic acid demonstrated an increasing trend (see Table 5). Partial differential metabolites are shown in Table 5; the full contents can be reached by connecting with our team.

#### 3.2.8. Metabolic Pathways of Feces and Urine

Under the basis of analyzing the differential metabolites, two sets of data were put into the channel of the model organism together. The metabolic pathways of different metabolites were enriched and analyzed to identify the metabolic pathways with significant influence. Then the bubble diagram of the metabolic pathway is shown in Figure 8. Each ring in the diagram represents a different metabolic pathway produced by the metabolic pathway analysis, and the color of each circle represents the *P* value. The redder the color, the smaller the *P* value, the higher the significance, and the larger the corresponding −log (*P*) value. The size of the circle indicates the influence of this metabolic pathway. The larger the circle, the greater its impact. As depicted in Figure 8, if the ring is closer to the upper-right side of the diagonal line, the metabolic pathway is more likely to be sought.

In the analysis of fecal differential metabolic pathways, there were significant differences between metabolic pathways such as pantothenate and CoA biosynthesis, alanine, aspartate, and glutamate metabolism, vitamin B6 metabolism, and nicotinate and nicotinamide metabolism (see Figures 8(a)–8(c)).

In the analysis of urine differential metabolic pathways (see Figures 8(b)–8(d)), metabolic pathways such as alanine, aspartate and glutamate metabolism, nicotinate and nicotinamide metabolism, histidine metabolism, taurine and hypotaurine metabolism, and arginine and proline metabolism exhibited significant differences.

## 4. Discussion

The metabolic pathways coincide in positive and negative ion modes in the spleen-deficiency children and the healthy group. According to *P* < 0.05 and considerable impact values, three metabolic pathways with significant differences were screened: the tryptophan pathway, the cysteine and methionine pathway in positive ion mode, and the pentose phosphate pathway (PPP) in the negative ion mode. Highly connected differential metabolites such as adenine, xanthine, glucuronic acid, and quinic acid, which were with the metabolism changes in comparing two groups, will also be discussed below.

Adenine and xanthine were in the differential metabolites lists between the spleendeficiency and healthy groups. Adenine [29, 30] is a component of nucleic acids and an essential part of coenzymes such as ATP and CoA and can be obtained by the hydrolysis of nucleic acids. Its phosphate can stimulate leukocytosis and is used to prevent and treat leukopenia caused by various reasons. All types of white blood cells have different defensive and protective functions, and timely and sufficient white blood cells are beneficial to defense against diseases. Xanthine is a derivative of purine that is frequently used as a mild stimulant and bronchodilator [31], especially for treating asthma symptoms [32]. In our results, adenine and xanthine have been proven to be at abnormal levels, which may lead to many health problems. Both are transferred from purine, mainly from the food we eat. Therefore, we hypothesize that the disorder of adenine and xanthine may be caused by improper eating diet or insufficient intestinal absorption, causing children with spleen-deficiency to have low immunity, a sensitive constitution, and are prone to illnesses.

Quinic acid [33, 34] is closely related to human intestinal metabolism. Quinic acid contributes to the synthesis of tryptophan and nicotinamide in the gastrointestinal tract [35, 36]. Nicotinamide plays a role in the metabolism of sugar and protein and can improve the nutrition of humans and animals. Additionally, quinic acid can improve bile, promote digestion, and reduce fat accumulation [37]. According to the results, quinic acid content was higher in spleen-deficiency children's bodily excretions than in healthy ones. Therefore, all these functions mentioned above may be less active inside the spleen-deficiency children's bodies, perhaps leading to the disorder of fat and other energy metabolisms in them. Abnormal energy metabolisms can increase the risk of suffering from digestive system diseases and may cause children with this constitution to be depressed, prone to fatigue, puffy, or sluggish. In its free form, quinic acid is broadly abundant in plants and can accumulate in copious amounts in coffee, tea, and certain fruits [33]. Because of the active efflux mechanism, the intestinal absorption of quinic acid is generally low [35]. Thus, we inferred that the quinic acid disorder of spleen-deficiency children might be caused by its lower intake and absorption, which may be related to eating diet and intestinal function.

Tryptophan has three metabolic pathways in the human intestine [38, 39]. Approximately 90% of tryptophan is converted into dog urine ammonia, 5% is directly metabolized by intestinal flora, and about 3% is transferred to 5-HT. As the results showed, children with spleen-deficiency have functional disorders in tryptophan metabolism, and those transfers may be increased or decreased. And tryptophan plays an essential role in intestinal immune tolerance and maintaining the balance of intestinal flora. Its metabolites also affect numerous intestinal functions such as barrier, peristalsis, digestion and absorption, secretion, and immunity [40]. Simultaneously, several studies have demonstrated a clear connection between tryptophan and oxidative stress [41–45]. When the tryptophan metabolism disorder in spleen-deficiency children appears, the producing process of dog urine ammonia, 5-HT may be disturbed, and the oxidative stress may be stimulated severely. All the changes may lead to frequent intestinal symptoms such as anorexia and diarrhea and affect mental factors like mood and sleep. Tryptophan [46] mainly comes from the body's initial protein or daily food; people can increase the body's tryptophan contents by taking particular food. Therefore, eating habits may affect the tryptophan metabolism in spleen-deficiency children, making them susceptible to numerous diseases, especially digestive diseases.

According to the results, children with spleen-deficiency had cysteine and methionine metabolism disorders, while cysteine and methionine benefit the human body. Cysteine plays a significant role in glutathione synthesis, increases oxidative stress in malnourished children, and reduces cysteine levels [47]. Methionine [48] is the raw material for synthesizing protein and cystine. Therefore, it positively affects the animal skeletal muscle development and the growth and development of embryos or offspring. As a functional essential amino acid in animals, methionine has positive effects on regulating animal physiological functions, antioxidant capacity, immune function, and intestinal health [49]. Methionine can also affect the digestion and absorption functions of the intestinal tract by improving the development of intestinal mucosal structure and boosting the activity of intestinal enzymes [50]. Cysteine content decreases when metabolic disorder happens, affecting children's growth and immunity. Compared with healthy children, the slow growth and poor immune ability of children with spleen-deficiency may be caused by the metabolic disorder of cysteine and methionine. Previous research [51] also showed that the methionine content in the serum of malnourished children was low, which is consistent with the results of this experiment. Cysteine and methionine mainly come from in vitro food intake. The difference in the pathway may be caused by the lack of relevant input in the diet of children with spleen-deficiency, which may be related to family eating habits and personal preferences.

The main characteristics of PPP are the direct decarboxylation and oxidative dehydrogenation of glucose, while glucuronic acid is one of the products [52]. In the experimental results, glucuronic acid levels in spleen-deficiency children presented a downtrend, indicating that the function of this approach is insufficient. PPP is a common pathway of sugar catabolism in animals, plants, and microorganisms [53]. Regular operation of PPP can help organisms transform nutrients from the external environment into substances. However, PPP is nearly lacking in the skeletal muscles of animals, while most glucose is decomposed through this pathway in adipose tissue, mammary glands, and the adrenal cortex [54]. In vivo, the pentose phosphate pathway provides energy and various raw materials for anabolism [55]. There may be a positive correlation between thin children with spleen-deficiency and PPP dysfunction. Those children have less fat to carry on the process of PPP. Meanwhile, the lack of PPP causes their abnormal energy metabolism and low physical function, which can explain why spleen-deficiency children are less energetic and less robust than healthy children. The source of this metabolic disorder may be related to their poor genes, digestion, and absorption.

## 5. Conclusion

The results showed that the metabolism condition varies between children with spleen-deficiency and healthy children. The children's spleen-deficiency constitution might result from disorders in tryptophan metabolism, cysteine and methionine metabolism, and pentose phosphate metabolism. These metabolism problems might be due to factors such as diet, personal preferences, and genes, leading to various symptoms. Setting up a specialized life and diet plan or choosing a therapy conducive to improving metabolism may improve this situation. Future researchers can explore more aspects of children with spleen-deficiency to create drugs and therapies to improve their body condition based on more results. Nevertheless, our study's sample size was small, and the study duration was not long. More studies are required to verify the conclusion of this experiment in the future.

## Figures and Tables

**Figure 1:** Process of the experiment.

**Figure 2:** Ion map (the left figures are results of the spleen deficiency group, while the right ones belong to healthy group. Results of (a) feces under positive ion mode; (b) feces under negative ion mode; (c) urine under positive ion mode; (d) urine under negative ion mode.

**Figure 3:** PCA score chart. Results of (a) feces under positive ion mode; (b) urine under positive ion mode; (c) feces under negative ion mode; (d) urine under negative ion mode.

**Figure 4:** PLS-DA score chart. Results of (a) feces under positive ion mode; (b) urine under positive ion mode; (c) feces under negative ion mode; (d) urine under negative ion mode.

**Figure 5:** Cross-validation chart of PLS-DA model. Results of (a) feces under positive ion mode; (b) urine under positive ion mode; (c) feces under negative ion mode; (d) urine under negative ion mode.

**Figure 6:** VIP diagram of PLS-DA. Results of (a) feces under positive ion mode; (b) urine under positive ion mode; (c) feces under negative ion mode; (d) urine under negative ion mode.

**Figure 7:** Heatmap analysis. Results of (a) feces under positive ion mode; (b) urine under positive ion mode; (c) feces under negative ion mode; (d) urine under negative ion mode.

**Figure 8:** Metabolic pathways of feces and urine. Results of (a) feces under positive ion mode; (b) urine under positive ion mode; (c) feces under negative ion mode; (d) urine under negative ion mode.

**Table 1:** Symptom lists of children with spleen-deficiency.

Names	Gender	Age (y)	Main symptoms	Accompanied symptoms
Zeng	M	6	Diarrhea, poor appetite, and sallow yellow complexion	Mild anemia
Li	M	5.5	Incomplete defecation and puffiness	Spontaneous sweating and mild anemia
Shu	M	5	Poor appetite, sallow yellow complexion, and incomplete defecation	Mild edema
Tang	M	4.5	Incomplete defecation, poor appetite, and wan complexion	Dark around the eyes
Tong	M	4.5	Puffiness and poor appetite	Mild edema and abdominal discomfort
Yang	F	4.1	Puffiness, sallow yellow complexion, and diarrhea	Mild edema, finger-licking, and salivation
Wu	F	4	Poor appetite, diarrhea, and emaciation	Hyperhidrosis, mild edema, limb weakness, and fatigue
Liu	F	4	Incomplete defecation, emaciation, and sallow yellow complexion	Faint finger venules and weak pulse and limb weakness and fatigue
Chen	M	4	Poor appetite, emaciation, wan complexion, and diarrhea	Limb weakness and fatigue
Chen	M	3	Diarrhea, wan complexion, and poor appetite	Abdominal discomfort and opening eyes while sleeping
He	M	3	Incomplete defecation and sallow yellow complexion	Spontaneous sweating, finger-licking, and salivation
Deng	F	3	Puffiness and fat tongue with teeth marks	Finger-licking and salivation and weak pulse
Tang	M	3	Diarrhea and poor appetite	Mild anemia, faint finger venules, and weak pulse
Guo	M	2.7	Diarrhea, emaciation, and poor appetite	Limb weakness and fatigue, faint finger venules
Liu	F	2.5	Diarrhea, sallow yellow complexion, and light tongue with greasy coating	Finger-licking and salivation and limb weakness and fatigue
He	M	2.1	Poor appetite, incomplete defecation, and wan complexion	Hyperhidrosis and mild edema
Fang	F	2	Poor appetite, incomplete defecation, and sallow yellow complexion	Opening eyes while sleeping and limb weakness and fatigue
Xiong	F	2	Diarrhea and poor appetite	Spontaneous sweating and mild anemia
Ni	M	1.5	Incomplete defecation and emaciation	Dark around the eyes, mild anemia, and limb weakness and fatigue
Tan	F	1	Diarrhea, poor appetite, and puffiness	Abdominal discomfort, faint finger venules, and weak pulse

**Table 2:** Chromatographic gradient.

Time (min)	Aqueous solution (liquid A)	Organic phase (liquid B)
0.0	90	10
1	90	10
13	2	98
18	2	98
18.5	90	10
20	90	10

**Table 3:** Mass spectrometry condition.

Parameter mass spectrometry	Parameter setting
Scanning mode	Separate scanning of positive and negative ions
Detection mode	Full mass/dd-MS2
Resolution	70000 (full mass); 17500 (dd-MS2)
Electrospray voltage	3.8 kV (positive); 3.2 kV (negative)
Capillary temperature	300°C
Sheath gas flow rate	40 Arb
Atomizer temperature	350°C

**Table 4:** Basic information comparison and clinical manifestation scores.

Groups	Gender (*n*)		Age (y)	Height (cm)	Weight (kg)	Face scores	Appetite scores	Sleep scores	Feces scores	Total scores
	M	F								
Healthy group	14	3	4.62 ± 1.27	95.30 ± 10.38	13.53 ± 2.10	1.00 ± 0.71	1.18 ± 0.73	0.47 ± 0.51	1.35 ± 0.79	4.00 ± 1.41
Spleen deficiency group	15	5	3.52 ± 1.35	94.45 ± 14.08	13.40 ± 3.74	2.10 ± 1.02^*∗*^	2.85 ± 1.08^*∗*^	1.40 ± 0.75^*∗*^	3.40 ± 1.31^*∗*^	9.70 ± 2.36^*∗*^

*Note*: compared with the healthy group, ^*∗*^means *P* < 0.05.

**Table 5:** Partial differential metabolites.

Names	VIP value	Fold change	*P* value	Average Rt (min)	Average (Mz)
Phosphatidylethanolamine lyso 18	1.9162	0.21446	0.10062	12.516	478.293
Alpha-phosphatidylethanolamine	1.8416	0.5076	0.21686	18.187	714.5065
Gluconic acid	1.8396	0.65788	0.58135	0.945	195.0503
Glutamic acid	1.8212	0.18241	0.085912	0.932	146.0446
Adenine	1.7725	6.0284	0.037128	1	134.0459
Aspartate	1.7482	1.5391	0.14615	0.851	132.0291
Glucuronic acid	1.7199	0.25446	0.0011781	0.898	193.0349
Threonine	1.688	0.81897	0.1156	0.875	118.0496
Xanthine	1.5756	0.30522	0.0040358	2.84	283.0687
Tryptophan.1	1.4066	0.4005	0.16809	5.067	203.0823
Fructose-6-phosphate	1.262	2.5851	0.094444	8.581	259.0246
Inosine	2.3652	0.32949	0.40494	1.84	269.08716
Diethanolamine	2.1253	4.69	0.23752	0.829	106.08647
Flufenacet ESA	1.9551	0.37409	0.28362	4.541	276.06921
Bisphenol A	1.7267	0.21512	0.12064	8.278	229.12183
Leucine	1.5922	0.97408	0.51278	0.855	132.10173
Indole-3-acetaldehyde	1.4689	0.32105	0.034672	7.041	158.0603
3-formylindole	1.5717	4.1966	0.021374	6.237	146.05991
4-methyl-5-thiazole-ethanol	1.5958	3.9271	0.037101	4.048	144.04787
5-hydroxy indole-3-acetic acid	1.5595	4.1977	0.042846	6.185	192.06531
Phenylalanine	1.5123	2.5864	0.70843	9.852	166.08578

## Data Availability

The data used in this study are available from the corresponding author upon request.

## References

[1] Jeong B. Y. (2022). Comparisons of working conditions and health-related problems between older male and female crop farmers. *Work*.

[2] Ogunniyi M. O., Commodore-Mensah Y., Ferdinand K. C. (2021). Race, ethnicity, hypertension, and heart disease: JACC focus seminar 1/9. *Journal of the American College of Cardiology*.

[3] Amezcua L., McCauley J. L. (2020). Race and ethnicity on MS presentation and disease course. *Multiple Sclerosis Journal*.

[4] Liang X., Wang Q., Jiang Z. (2020). Clinical research linking Traditional Chinese Medicine constitution types with diseases: a literature review of 1639 observational studies. *Journal of Traditional Chinese Medicine*.

[5] Wang Q. (2021). Reconsideration of the three key scientific issues of TCM constitution and its prospect: speech at the 19th academic annual meeting of the TCM Constitution Branch, China Association of Chinese Medicine. *Journal of Beijing University of Traditional Chinese Medicine*.

[6] Dong S., Zhao Z., Li W. (2022). Research on translation of Chinese medicine constitution (tizhi) academic terms: based on memetics and delphi method. *Evidence-based Complementary and Alternative Medicine*.

[7] Wang H. R., Yu N., Liu Z., Zhai S. Q. (2017). Comparison of constitutionology between huangdi neijing and modern TCM. *China Journal of Traditional Chinese Medicine and Pharmacy*.

[8] Cen H., Wang Q. (2007). Multiple linear regression analysis of body constitution and sub-health of TCM. *Traditional Chinese Medicinal Research*.

[9] Zhang Y., Fu J., Zhou Z., Zhang Y., Chen Y., Song A. (2022). Exploring the relationship between allergic rhinitis and constitution based on the ‘traditional Chinese medicine constitution theory. *Evidence-based Complementary and Alternative Medicine*.

[10] Lai N. S., Lu M. C., Chang H. H. (2021). Association of traditional Chinese medicine body constitution and health-related quality of life in female patients with systemic lupus erythematosus: a cross-sectional study. *Evidence-based Complementary and Alternative Medicine*.

[11] Pan P. G., Xu L. P., Zhou J. L., Wang X., Tian H. (2010). Identification of common TCM constitutions of children aged from 0 to 6 years old. *New Chinese Medicine*.

[12] Liu X. (2012). Research status on classification and determination of constitution in TCM. *The First International Forum on Constitution Theory —— A Collection of Papers from the 10th Annual Meeting of the Chinese Society of Traditional Chinese Medicine*.

[13] Qu J. L., Di E. F. (2022). Test and analysis of children’s traditional Chinese medicine constitution evaluation system. *Journal of Practical Traditional Chinese Internal Medicine*.

[14] Wang Q. H., Yan J. T. (2021). Research on the mechanism of manipulation in the treatment of functional dyspepsia in children. *Chinese Manipulation and Rehabilitation Medicine*.

[15] Cheng W. W., Wang L., Feng Y. L., Jing X. P., Liu H. F. (2022). Effect of shenling baizhusan on electrogastrogram in children with spleen deficiency diarrhea. *Chinese Journal of Experimental Traditional Medical Formulae*.

[16] Hang Y. H., Tian C. X. (2021). Clinical curative effect analysis of modified banxia xiexin decoction in treating children’s functional constipation of spleen deficiency type. *The Journal of Medical Theory and Practice*.

[17] Zhang J. J., Ye J. (2017). Professor YE’s clinical experiences for dwarfism treatment based on spleen-insufficiency constitution related theory. *Journal of Zhejiang Chinese Medical University*.

[18] Long M., Xu L. (2022). Discussion on the significance of prevention and treatment of childhood asthma based on intestinal flora theory of spleen deficiency. *Acta Chinese Medicine and Pharmacology*.

[19] Bauermeister A., Mannochio-Russo H., Costa-Lotufo L. V., Jarmusch A. K., Dorrestein P. C. (2022). Mass spectrometry-based metabolomics in microbiome investigations. *Nature Reviews Microbiology*.

[20] Du X. Z., Wang J. H., Zhang X. H. (2016). Influence of heat-reinforcing needling on expression of plasma atp 50 mRNA and atp 6V1B2 mRNA in patients with rheumatoid arthritis of windcold-damp retention type. *Acupuncture Research*.

[21] Bao X. H., Bao L. M., Xiang C., Gerile S., Qiqige S., Xie Y. L. (2022). Metabolic characterization of the badagan constitution in Mongolian medicine by ultrahigh-performance liquid chromatography/quadrupole time-of-flight mass spectrometry/MS. *World Journal of Traditional Chinese Medicine*.

[22] Chen Y., Wu Y., Yao H. (2018). miRNA expression profile of saliva in subjects of yang deficiency constitution and yin deficiency constitution. *Cellular Physiology and Biochemistry*.

[23] (2000). Diagnosis criteria of spleen deficiency Syndrome in children. *Chinese Journal of Integrated Traditional and Western Medicine*.

[24] Liao P. D. (2016). *Pediatric Massage*.

[25] Wang Z. C., Wang X. N. (2008). Discussion about the theoretical basis of constitution and sub- health prevention and treating. *Chinese Archives of Traditional Chinese Medicine*.

[26] (2009). The Ministry of Health issued a reference standard for the growth and development of children under 7 years old. *China Journal Prevention Control Chronic Disease*.

[27] Zhu W. F. (2018). *Diagnostics of Traditional Chinese Medicine*.

[28] Zheng X. Y. (2002). *Guidance Principle of Clinical Study on New Drug of Traditional Chinese Medicine*.

[29] Tsukahara T., Sahara Y., Ribeiro N. (2021). Adenine nucleotide translocase 2, a putative target protein for 2-carba cyclic phosphatidic acid in microglial cells. *Cellular Signalling*.

[30] Ding J. L., Wei X. X., Ren X. F. (2015). Optimization of extraction technology for adenine from oviductus ranae by central composite design/response surface methodology. *Practical Pharmacy and Clinical Remedies*.

[31] Flores S., Culichia C. N., Villarreal E. G., Savorgnan F., Checchia P. A., Loomba R. S. (2020). Xanthine derivatives for kidney protection in the critically ill pediatric population: a systematic review. *Journal of Pediatric Intensive Care*.

[32] Yang Y. Y. (2017). *The Relationship between the Anti-nociception of Propentofylline on Rats of Incisional Pain and MKP-1/p-P38*.

[33] Naranjo Pinta M., Montoliu I., Aura A. M., Seppanen-Laakso T., Barron D., Moco S. (2018). In Vitro gut metabolism of [U-^13^ C]-quinic acid, the other hydrolysis product of chlorogenic acid. *Molecular Nutrition & Food Research*.

[34] Heikkilä E., Hermant A., Thevenet J. (2019). The plant product quinic acid activates Ca^2+^ -dependent mitochondrial function and promotes insulin secretion from pancreatic beta cells. *British Journal of Pharmacology*.

[35] Mortelé O., Jörissen J., Spacova I., Lebeer S., van Nuijs A. L. N., Hermans N. (2021). Demonstrating the involvement of an active efflux mechanism in the intestinal absorption of chlorogenic acid and quinic acid using a Caco-2 bidirectional permeability assay. *Food & Function*.

[36] Hong Z. C. (2019). *Component Analysis and Metabolomics Study of Fufang Kushen Decoction against Ulcerative Colitis*.

[37] Clifford M. N., Kerimi A., Williamson G. (2020). Bioavailability and metabolism of chlorogenic acids (acyl- quinic acids) in humans. *Comprehensive Reviews in Food Science and Food Safety*.

[38] Hyland N. P., Cavanaugh C. R., Hornby P. J. (2022). Emerging effects of tryptophan pathway metabolites and intestinal microbiota on metabolism and intestinal function. *Amino Acids*.

[39] Licari A., Fuchs D., Marseglia G., Ciprandi G. (2019). Tryptophan metabolic pathway and neopterin in asthmatic children in clinical practice. *The Italian journal of pediatrics*.

[40] Comai S., Bertazzo A., Brughera M., Crotti S. (2020). Tryptophan in health and disease. *Advances in Clinical Chemistry*.

[41] Leonardi S., Pecoraro R., Filippelli M. (2014). Allergic reactions to foods by inhalation in children. *Allergy and Asthma Proceedings*.

[42] Wigner P., Czarny P., Galecki P., Su K. P., Sliwinski T. (2018). The molecular aspects of oxidative & nitrosative stress and the tryptophan catabolites pathway (TRYCATs) as potential causes of depression. *Psychiatry Research*.

[43] Xu K., Liu H., Bai M., Gao J., Wu X., Yin Y. (2017). Redox properties of tryptophan metabolism and the concept of tryptophan use in pregnancy. *International Journal of Molecular Sciences*.

[44] Zou M. H., Liu D., Song P., Zou M. H. (2015). Tryptophan-kynurenine pathway is dysregulated in inflammation, and immune activation. *Frontiers in Bioscience*.

[45] Zhuravlev A. V., Vetrovoy O. V., Savvateeva-Popova E. V. (2018). Enzymatic and nonenzymatic pathways of kynurenines’ dimerization: the molecular factors for oxidative stress development. *PLoS Computational Biology*.

[46] Coma S., Bertazzo A., Brughera M., Crotti S. (2020). Tryptophan in health and disease. *Advances in Clinical Chemistry*.

[47] Badaloo A., Hsu J. W., Taylor-Bryan C. (2012). Dietary cysteine is used more efficiently by children with severe acute malnutrition with edema compared with those without edema. *American Journal of Clinical Nutrition*.

[48] Olsen T., Øvrebø B., Turner C., Bastani N. E., Refsum H., Vinknes K. J. (2021). Effects of short-term methionine and cysteine restriction and enrichment with polyunsaturated fatty acids on oral glucose tolerance, plasma amino acids, fatty acids, lactate and pyruvate: results from a pilot study. *BMC Research Notes*.

[49] Feng Y., Yang L., Zhu Y. W., Wang W. C. (2019). Methionine regulates the major physiological functions of animals. *Scientia Sinica Vitae*.

[50] Yu Y. M., Liu D., Zhang B. K. Intestinal barrier function and nutritional regulation of poultry.

[51] Elango R. (2020). Methionine nutrition and metabolism: insights from animal studies to inform human nutrition. *Journal of Nutrition*.

[52] Hambardikar V., Guitart-Mampel M., Scoma E. R. (2022). Enzymatic depletion of mitochondrial inorganic polyphosphate (polyP) increases the generation of reactive oxygen species (ROS) and the activity of the pentose phosphate pathway (PPP) in mammalian cells. *Antioxidants*.

[53] Stincone A., Prigione A., Cramer T. (2015). The return of metabolism: biochemistry and physiology of the pentose phosphate pathway. *Biological Reviews*.

[54] Riganti C., Gazzano E., Polimeni M., Aldieri E., Ghigo D. (2012). The pentose phosphate pathway: an antioxidant defense and a crossroad in tumor cell fate. *Free Radical Biology and Medicine*.

[55] Ramos-Martinez J. I. (2017). The regulation of the pentose phosphate pathway: remember Krebs. *Archives of Biochemistry and Biophysics*.

